# Effect of Hematocrit Injury on the Survival Rate of Advanced Malignant Tumors and Its Clinical Significance

**DOI:** 10.1155/2022/4968754

**Published:** 2022-06-15

**Authors:** Lin Li, Weibin Wu, Mingdi Yin

**Affiliations:** ^1^Shaanxi Provincial Cancer Hospital Pathology Department, 710068, China; ^2^Shaanxi Provincial Cancer Hospital Transfusion Department, 710068, China; ^3^Shaanxi University of Chinese Medicine Faculty of Medicine and Technology Department of Laboratory, 710068, China

## Abstract

**Objective:**

To investigate the effect of logistic multivariate analysis on the survival rate of advanced malignant tumors and to evaluate the effect of erythrocyte storage injury on the survival rate of advanced malignant tumors and its clinical significance.

**Methods:**

A retrospective analysis was performed on 120 advanced cancer patients who received blood transfusion in Shaanxi Cancer Hospital from March 2018 to June 2019, and the risk factors for death were analyzed. A total of 72 advanced cancer patients admitted to hospital from March 2019 to June 2021 were included in the study. The patients with red blood cell transfusion storage time ≤ 14 d were the study group (*n* = 36), and the patients with red blood cell transfusion storage time > 14 d were the control group (*n* = 36). Compare the total efficiency of blood transfusion. The levels of Hb, erythrocyte count, hematocrit (HCT), blood oxygen saturation (SPO2), creatinine (Cr), erythrocyte deformability index, whole blood, erythrocyte, and hemoglobin before and after blood transfusion were compared, and the adverse reactions of blood transfusion were recorded.

**Results:**

Dyspnea and delirium were significantly associated with patient survival time (*P* < 0.05). Red blood cell storage time ≤ 14 days, Lym% < 12%, lactate dehydrogenase (LDH) > 500 U/L, and ALB < 30 g/L were significantly correlated with survival time. Karnofsky performance status (KPS) < 30, delirium, LDH > 500 U/L, and albumin (ALB) < 30 g/L were independent influencing factors of survival (*P* < 0.05). The overall effective rate of the research group was higher (*P* < 0.05). The incidence of adverse reactions in the study group was lower (*P* < 0.05). The levels of Hb, red blood cell count, and HCT in the study group were higher (*P* < 0.05). Compared with the control group, the SPO2 level and the red blood cell deformability index were higher in the study group (*P* < 0.05). After blood transfusion, the level of (diphosphoglycerate) DPG in the study group was higher than that in the control group (*P* < 0.05). The length of hospital stay in the study group was significantly shortened (*P* < 0.05). The nosocomial infection rate and case fatality rate in the study group were significantly reduced (*P* < 0.05).

**Conclusion:**

Red blood cell storage time ≤ 14 d, LYM% < 12%, LDH > 500 U/L, and ALB < 30 g/L are all significantly correlated with survival time. KPS < 30, delirium, LDH > 500 U/L, and ALB < 30 g/L were independent factors for survival (*P* < 0.05). Transfusion of red blood cells stored for ≤14 days in patients with advanced malignant tumors can significantly increase the effective infusion rate, improve anemia status, shorten hospital stay, and reduce mortality and risk of nosocomial infection and is worthy of clinical promotion.

## 1. Introduction

Since 2010, tumor has become the “number one killer” endangering the health of people [1]. In recent years, its morbidity and mortality have increased year by year. Whether in urban or rural areas, cancer is the primary public health problem that we must face. Malignant tumor anemia is a common complication of malignant tumor patients. According to statistics, about 50% of malignant tumor patients develop anemia, and the incidence of anemia is as high as 90% in patients with advanced malignant tumors and patients receiving radiotherapy or chemotherapy or concurrent radiotherapy and chemotherapy, further increasing the degree of hypoxia of tumor cells [2]. Cancerous anemia will not only reduce the quality of life of patients but also reduce the therapeutic effect of cancer, thus indirectly reducing the survival rate of patients. Cancerous anemia may be one of the independent prognostic factors affecting the survival of cancer patients, so it is necessary for cancer patients to receive blood transfusion [3].

Hemoglobin is an important oxygen-carrying tool in the human body. 1.5% to 2.0% of the oxygen in the blood exists in a physical state, and most of the oxygen binds to hemoglobin, and the decrease in the concentration of hemoglobin in the blood leads to tissue hypoxia, which further increases the percentage of hypoxic cells in tumor tissue [2, 3]. The killing effect of tumor radiotherapy depends to a large extent on the oxygen content of tumor cells, which can be said to be the strongest radiosensitizer [4]. In clinical findings, hemoglobin concentration before and after radiotherapy had an effect on local control rate, survival rate with or without recurrence, and overall survival rate [4]. Blood transfusion can quickly correct anemia. Although blood transfusion is widely adopted in clinic, our blood safety assessment is often limited to blood infectious diseases and adverse reactions of blood transfusion, ignoring the effect of blood quality on the safety and effectiveness of blood transfusion. At present, the storage time of suspended red blood cells in China is up to 35 days, and the quality control requirements for whole blood and component blood are carried out in accordance with GB18469-2012, but except for the detection of infectious diseases, all other requirements are recommended. For suspended red blood cells, the standard specifies the appearance, volume, and hematocrit and hemoglobin content of blood and requires that the result of bacterial culture is negative and the hemolysis rate at the end of storage is less than 0.8%. Hemolysis rate = (1 − hematocrit) × supernatant free hemoglobin concentration/total hemoglobin concentration × 100% [4, 5]. Although these indexes are easy to detect, they cannot reflect the changes of erythrocyte survival rate and cell morphology, nor can they reflect the changes of cell activity, oxygen-carrying capacity and agglutination function. The safety and effectiveness of blood that meets this standard for clinical patients have not been confirmed by large-scale clinical trial data. In addition, the red blood cells for clinical use need to be transported from the blood station to the hospital blood bank and stored in the blood bank for a period of time, this process will cause erythrocyte destruction, and the final hemolysis rate of red blood cells imported into the patient at the end of storage is also unknown [6]. It can be noticed that the current quality control standard for blood cannot guarantee the survival of 90% of infused red blood cells within 48 hours, and even blood with a survival rate of much less than 70% of red blood cells will be considered qualified, but the infusion of dead and dysfunctional red blood cells will only have a negative impact on the patients [7].

The accurate prediction of the survival time of patients with end-stage malignant tumor can not only give patients and their families a full understanding of the disease but also provide some guidance for medical workers in the choice of treatment [8]. Some scholars have indicated that the factors affecting the survival of patients with end-stage malignant tumors are closely related to the main clinical symptoms and hematological indicators of patients [8, 9]. Some scholars have also screened out the independent factors that affect the survival time of end-stage malignant tumors, but these methods cannot be widely adopted because of the influence of survival time, population, and other factors [10, 11]. Therefore, at present, a unified standard has not been established on the factors affecting the survival of patients with end-stage malignant tumors. The purpose of this study is to analyze the blood-related indexes that affect the survival of patients with end-stage malignant tumors and to find out the factors that have a significant impact on the survival time, so as to provide a scientific basis for better selection of correct and appropriate treatment.

## 2. Patients and Methods

### 2.1. General Information

One hundred and twenty patients with advanced tumor treated by blood transfusion in Shaanxi Cancer Hospital from March 2018 to June 2019 were analyzed retrospectively. All patients were advanced malignant tumor patients who could not tolerate surgery, radiotherapy, and chemotherapy and received the best supportive treatment; general information is indicated in Table 1. Another 72 patients with advanced cancer admitted from March 2019 to June 2021 were enrolled as the study object. The patients with red blood cell transfusion storage time ≤ 14 days were enrolled as the study group (*n* = 36), and the patients with red blood cell transfusion storage time > 14 days were enrolled as the control group (*n* = 36). There were 16 males and 20 females in the study group, with an average age of 61.15 ± 23.42 years, while in the control group, there were 18 males and 18 females, with an average age of 60.92 ± 23.26 years. This study was permitted by the Medical Ethics Association of our hospital, and all patients noticed informed consent.

Selection criteria are as follows: (1) regardless of gender, patients with end-stage malignant tumors who could not receive relevant active antitumor therapy were admitted to hospital to receive the best palliative treatment; (2) without cognitive, language, and intellectual impairment and having basic reading and writing ability; (3) agree to follow-up and be able to accept and answer telephone followers; and (4) complete clinical data.

Exclusion criteria are as follows: (1) refuse to participate; (2) patients cannot obey treatment and late rehabilitation physiotherapy because of mental and psychological diseases; and (3) patients with incomplete clinical data.

### 2.2. Treatment Methods

Clinical data include general information of patients, main clinical symptoms, and hematological indicators. The general information and clinical symptoms were collected on admission, and the hematological indexes were collected in the morning on the second day of admission. General information includes age, sex, diagnosis, location of primary malignant tumor, number and location of metastatic foci, previous treatment methods, and Karnofsky performance status (KPS); clinical symptoms include pain, nausea and vomiting, dyspnea, cough, anorexia, abdominal distension, constipation, diarrhea, insomnia, looking forward, bleeding, cachexia, fever, and weight loss. The main hematological indexes include white blood cell (WBC), hemoglobin (Hb), lymphocyte percentage (Lym%), neutrophil percentage (Neu%), platelet (PLT), total bilirubin (TBIL), alkaline phosphatase (ALP), glutamic pyruvic transaminase (GPT), glutamic oxaloacetic transaminase (GOT), lactate dehydrogenase (LDH), albumin (ALB), serum potassium, serum sodium, and serum calcium. Survival is defined as the time from admission to death (accurate to days). It is evaluated by clinicians in strict accordance with the standards required by the Technical Specification for Clinical Blood Transfusion, and blood transfusion treatment is given after signing the consent form for blood transfusion.

### 2.3. Observation Index

(1) To compare the incidence of adverse transfusion reactions; (2) to compare the levels of Hb before and after transfusion and to calculate the Hb recovery rate and the total effective rate of transfusion; (3) to compare the changes of hematocrit (HCT), blood oxygen saturation (SPO2), red blood cell count, and creatinine (Cr) before and after transfusion; (4) the Hb level of patients was detected 24 hours after red blood cell transfusion. Hb recovery rate = Wt × *V* × (postinfusion Hb level − pre − infusion Hb level); the total input Hb is ×100%, where Wt is the patient's body mass (kg) and *V* is the blood volume per kilogram of body mass; adults are 0.07 L/kg, and infants are 0.08 L/kg. The calculation of the total amount of input Hb: the total amount of Hb per unit of red blood cells (calculated by 24 g/U) × the amount of input erythrocytes (U). According to the Hb recovery rate, >79% is obviously effective, >49% is more effective, ≥20% is partially effective, and <20% is invalid. Total effective rate of blood transfusion = obvious effective rate + more effective rate.

### 2.4. Statistical Analysis

The data were processed by SPSS16.0 statistical software, and the survival time was calculated by the Kaplan-Meier method. The related factors were analyzed by univariate analysis and tested by log-rank method. The Cox regression model was adopted to analyze the significant factors in univariate analysis, and the prognostic factors with independent significance were screened out. The counting data are presented as cases or percentage, using *χ*^2^ test, and the measurement data in accordance with normal distribution are presented as *x* ± *s*, using *t*-test. The difference exhibited statistically significant (*P* < 0.05).

## 3. Results

### 3.1. General Data of 120 Dead Patients

First of all, we analyzed the general data of 120 dead patients. The average age of 120 dead patients was 63.15 ± 18.42 years old (24 to 93 years old). 51.67% (62 cases) of the patients were male. 81.22% of the patients had a definite pathological diagnosis, and the other patients were clinically diagnosed as stage IV advanced tumor. There were 21 cases of lung cancer (17.50%), 12 cases of breast cancer (10.00%), 52 cases of digestive system tumors (43.33%), 12 cases of gynecological tumors (10.00%), 8 cases of urinary system tumors (6.67%), and 15 cases of other tumors (12.50%). Fifty-seven patients (47.50%) had more than two distant metastases. The most common metastatic sites were liver (*n* = 45) and bone (*n* = 44). 64 cases (53.33%) had previously received surgery, 48 cases (40.00%) had received radiotherapy, and 71 cases (59.17%) had received chemotherapy. All the results are indicated in Table 1.

### 3.2. Overall Survival of Patients with Advanced Malignant Tumor

We analyzed the overall survival of patients with advanced malignant tumors. The average survival time of 120 patients who died was 26 days (1-127 days, 95%Cl: 22-28), and the median survival time was 17 days (95%Cl: 13-19). 14 patients died within 1 day of admission, and the 1-week survival rate was 70.11%. The 2-week survival rate was 52.76%, and the 4-week survival rate was 32.1%. All the results are indicated in Figure 1.

### 3.3. Univariate Analysis of Factors Affecting Survival in Patients with Advanced Malignant Tumor

We conducted a univariate analysis of the factors affecting the survival of patients with advanced malignant tumor. The results indicated that dyspnea and delirium were remarkably correlated with the survival time of patients (*P* < 0.05). Laboratory hematological indexes are more objective and operable than KPS and clinical symptoms. In this study, erythrocyte storage time (erythrocyte storage time means preservation time of infusion red blood cells) ≤ 14 days, Lym% < 12%, LDH > 500 U/L, and ALB < 30 g/L were remarkably correlated with survival time. All the results are indicated in Table 2.

### 3.4. Multivariate Analysis of Factors Affecting Survival Time of Patients with Advanced Malignant Tumor and Cox Regression Model

Seven factors obtained from univariate analysis were included in the enrolled variables of Cox, and multivariate analysis of Cox regression model indicated that KPS < 30, delirium, LDH > 500 U/L, and ALB < 30 g/L were independent influencing factors of survival (*P* < 0.05). All the results are indicated in Table 3.

### 3.5. Comparison of the Total Effective Rate

We compared the total effective rate. In the study group, 22 cases were obviously effective, 9 cases were more effective, 3 cases were partially effective, and 2 cases were invalid, and the excellent rate was 94.44%. In the control group, 19 cases were obviously effective, 7 cases were more effective, 2 cases were partially effective, and 8 cases were invalid, and the excellent rate was 77.78%. The total effective rate of the study group was higher (*P* < 0.05). All the results are indicated in Figure 2.

### 3.6. Comparison of Adverse Reactions of Blood Transfusion

We compared the adverse reactions of blood transfusion. In the study group, there were 1 case of fever and 2 cases of allergy. The incidence of adverse reactions was 8.33%. In the control group, there were 7 cases of fever and 6 cases of allergy. The incidence of adverse reaction was 36.11%. The incidence of adverse reactions in the study group was lower (*P* < 0.05). All the results are indicated in Figure 3.

### 3.7. Comparison of Hb Level, Erythrocyte Count, and HCT before and after Blood Transfusion

We compared the Hb level, red blood cell count, and HCT of patients before and after blood transfusion. Before blood transfusion, there exhibited no significant difference in Hb level, red blood cell count, and HCT (*P* > 0.05). After blood transfusion, the Hb level, red blood cell count, and HCT level of the two groups of patients were all increased. Compared between the two groups, the Hb level, red blood cell count, and HCT level of the study group were higher (*P* < 0.05). All results are indicated in Table 4.

### 3.8. Comparison of SPO2 Level, Cr Level, and Erythrocyte Deformation Index before and after Transfusion

We compared the levels of SPO2, Cr, and erythrocyte deformation index before and after blood transfusion. Before blood transfusion, there exhibited no significant difference in SPO2 level, Cr level, and erythrocyte deformation index (*P* > 0.05). After blood transfusion, the Cr levels in both groups decreased, but there was little change between the observation group and the control group, and the difference exhibited was not statistically significant (*P* > 0.05). After blood transfusion, the SPO2 level and erythrocyte deformation index increased. Compared between the two groups, the SPO2 level and erythrocyte deformation index of the study group were higher (*P* < 0.05). All the results are indicated in Table 4.

### 3.9. Comparison of (Diphosphoglycerate) DPG Levels of Whole Blood, Red Blood Cells, and Hemoglobin before and after Blood Transfusion

We compared the levels of SPO2, Cr, and erythrocyte deformation index before and after blood transfusion. Before transfusion, there exhibited no significant difference in the levels of whole blood, red blood cells, and hemoglobin 2mazel DPG (*P* > 0.05). After blood transfusion, the levels of whole blood, erythrocytes, and hemoglobin 2,3-DPG in the two groups were all increased. Comparison between the two groups indicated that the levels of whole blood, erythrocytes, and hemoglobin 2,3-DPG in the study group were higher (*P* < 0.05). All results are indicated in Table 4.

### 3.10. Comparison of Hospital Stay, Nosocomial Infection Rate, and Mortality after Blood Transfusion

We compared the hospitalization time, hospital infection rate, and mortality after blood transfusion. The average hospital stay was 18.36 ± 3.31 days in the study group and 32.87 ± 2.18 days in the control group; the hospitalization time of the study group was remarkably shorter (*P* < 0.05). Among them, 3 cases died in the study group, 1 case had nosocomial infection, 12 cases died in the control group, and 10 cases occurred nosocomial infection. The nosocomial infection rate and mortality in the study group were remarkably lower (*P* < 0.05).

## 4. Discussion

The incidence of anemia in patients with advanced cancer is high, which is the main group of patients who need blood transfusion [12]. Such patients are generally older, having low immune function, often accompanied by metabolic disorders and abnormal blood coagulation, and may be more sensitive to changes in blood quality. The effect of blood quality on patients comes from the “storage damage” of red blood cells; that is, with the extension of storage time, the concentration of 2,3-diphosphoglyceric acid, the metabolism level of nitric oxide, and the fragility of cell membrane and cell adhesion decrease with the extension of storage time. These changes lead to the decrease of oxygen-carrying capacity and increase the risk of hemolysis and blood agglutination, meanwhile, in cell maintenance solution. The concentrations of free hemoglobin, free iron, potassium, and inflammatory mediators increased [13]. This change in red blood cells may increase the incidence of adverse reactions and in-hospital mortality. The storage damage of red blood cells is closely related to the internal energy metabolism of red blood cells. Because there are no mitochondria in red blood cells relying entirely on glycolysis to obtain energy, the lactic acid produced in the process of glycolysis will reduce the internal pH value of cells, thus reducing the metabolic level of cells and reducing the production of ATP, resulting in a decrease in the level of phosphoprotein phosphorylation and loss of deformability of cell membrane. The decrease of ATP level will lead to the decrease of 2,3-diphosphoglyceric acid synthesis, and the decrease of pH value and the concentration of 2Magne3-diphosphoglyceric acid will shift the oxygen dissociation curve of hemoglobin to the left, resulting in the decrease of oxygen-carrying function of the cells [14]. ATP is also an agonist of NO synthase. NO and hemoglobin in erythrocytes combine to form SNOHb and Hb (Fe~II) NO, which participate in the transport and metabolism of NO. The decrease of ATP also affects the ion pump on the cell membrane, resulting in an increase in the level of K+ in stored blood. At present, some scholars mostly focus on the relationship between blood quality and adverse reactions of blood transfusion and the changes of blood physical and chemical indexes [15]. There are few clinical research data such as mortality, infection rate, incidence of complications, and average length of stay in hospital.

The effect of “storage injury” of red blood cells on patients has always been a hot issue in some clinical research, which may be related to the long shelf life of red blood cells abroad (42 days) [16]. In recent years, journals such as the New England Journal have reported a series of multicenter, large-scale clinical trials for different groups of patients to discuss the effects of erythrocyte storage injury on patients. These studies show that the effect of “old” red blood cells on patients is closely related to the types of diseases and the selection of indicators to evaluate the disease, and the conclusions of different diseases are quite different [16, 17]. When Koch et al. conducted a retrospective study of more than 6000 patients who received blood transfusion after cardiac surgery, they found that the incidence of serious postoperative complications and hospital death in patients with “old” red blood cells with preservation time of more than two weeks were remarkably higher than those with “fresh” red blood cells with preservation time less than two weeks. Another study of trauma patients found that mortality increased only in patients who received more than three units of “old” red blood cells within 24 hours [17]. For healthy volunteers, transfusion of “old” red blood cells only increased the risk of extravascular hemolysis and infection. In animal experiments, the infusion of a large number of “old” red blood cells remarkably increased the mortality of pneumonia model dogs and led to more severe lung injury [18]. Wang et al. conducted a meta-analysis of 21 studies and indicated that the transfusion of “stale” red blood cells remarkably increased the risk of death in patients [19]. However, other studies have indicated that there is no significant difference in the effect of transfusion of “stale” red blood cells and “fresh” red blood cells on patients. A randomized controlled trial conducted by Heddle et al. found that transfusion of “stale” or “fresh” RBCs did not affect in-hospital mortality in general inpatients [20]. Transfusion of “fresh” red blood cells also did not reduce patient mortality. There are also some diseases, and the research results of different institutions are completely opposite, which may be caused by the difference in the indicators they choose and the quality of blood preservation [21]. Although the American Blood Transfusion Association concluded in 2016 based on the results of 13 clinical trials that the current evidence is insufficient to prove that red blood cells during the shelf life will cause adverse events to patients, many researchers believe that “old” blood will adversely affect patients, while the American Blood Transfusion Association refers to these trials on a small scale, involving fewer diseases, one-sided evaluation indicators, flawed statistical methods, and a low level of evidence [22].

The subjects of this study were 120 patients with advanced malignant tumors who received palliative treatment. The primary tumors were of various locations; metastatic sites, numbers, and previous courses of the disease were different [23]. The study obtained a total of four independent factors affecting the survival and prognosis of patients, which is the same as some previous studies in this field, but also got new results worthy of attention. KPS is a clinical index to evaluate the general condition of tumor patients, not only as a reference index for the choice of treatment but also an important evaluation standard of curative effect. For patients with advanced malignant tumors, KPS has been confirmed for many times to have a significant correlation with survival [24]. It is worth noting that the KPS scoring process cannot rule out the subjective impression of clinicians. The acquisition of subjective impression is related to more clinical-related factors. However, this does not affect the prognostic value of KPS. Dyspnea is one of the common symptoms in patients with advanced malignant tumor, which is often caused by a variety of reasons [25]. Frequent and uncontrollable dyspnea is also the most important clinical symptom in patients with advanced malignant tumor, which is proved to be remarkably related to the survival and prognosis of advanced patients [26]. In this study, 30.00% (36 cases) of patients complained of dyspnea, and the survival time of these patients was remarkably shorter compared to patients without this symptom. It has been confirmed that the occurrence and degree of dyspnea are related to the decrease of Hb. However, this study did not confirm that the decrease of Hb is a prognostic factor. The correlation between them and their relationship with survival time are worthy of further study.

Delirium can be considered as a common syndrome of loss of consciousness in patients with advanced cancer [27, 28]. In this study, 20.83% of the patients indicated expectant symptoms on admission, which was similar to the 26.0%~44.0% reported [29]. Current studies believe that the emergence of delirium is the result of multiple clinical factors, including drugs, electrolyte disorders, endocrine disorders, hypoxemia, infection, paraneoplastic syndrome, intracranial metastasis, and dehydration [30], although the study reported that through appropriate intervention, the outlook of nearly 50% of patients with advanced cancer is reversible. However, the appearance of prospective symptoms is still an important factor affecting the survival prediction of patients with advanced cancer. Related studies have further optimized the existing survival prediction models according to whether patients have prospective symptoms or not. The correct evaluation of prospective symptoms and clinical intervention are worthy of further discussion.

Compared with clinical symptoms and KPS, laboratory indicators have better convenience, objectivity, and maneuverability. Red blood cell storage time and Lym% < 12% are important factors in the previous prediction models. Long storage time of red blood cells may adversely affect the survival time of patients, while the relatively high Lym indicates that the survival time is relatively optimistic. In this study, the red blood cell storage time of 57.50 patients was more than 14 days on admission, and the Lym% of 65.00% of the patients was less than 12%. Red blood cell storage time less than 14 days is a prognostic factor, but multivariate analysis does not support it as an independent prognostic factor. Lym% < 12% is an independent prognostic factor related to survival. The decrease of Lym% indicates the decrease of immunity, and its relationship with inflammatory factors such as anorexia (cachexia), weight loss, and C-reactive protein is worthy of further study.

Improving the anoxic state of patients' cells and tissues is the fundamental purpose of red blood cell transfusion. In this process, the quality changes of red blood cells during the whole storage period have an important impact on the therapeutic effect. Some studies have indicated that with the extension of storage time, the level of 2-diphosphoglyceric acid in red blood cells decreases and the morphology of red blood cells also changes. These changes may lead to the increase of red blood cell density, hardness, and permeability, thus affecting the transport of O_2_ and CO_2_ in red blood cells. In this study, 72 patients with advanced malignant tumor were enrolled as subjects to investigate the infusion effect of red blood cell storage time ≤ 14 days and >14 days. The results indicated that the total effective rate was compared. In the study group, 22 cases were obviously effective, 9 cases were more effective, 3 cases were partially effective, and 2 cases were invalid, and the excellent rate was 94.44%. In the study group, 19 cases were obviously effective, 7 cases were effective, 2 cases were partially effective, and 8 cases were invalid, and the excellent rate was 77.78%. The overall rate of effectiveness in the study group was higher (*P* < 0.05). In terms of the adverse reactions of blood transfusion, there were 1 example of fever and 2 cases of allergy in the study group, and the incidence of adverse reactions was 8.33%. In the control group, there were 7 cases of fever and 6 cases of allergy. The incidence of adverse reaction was 36.11%. The incidence of adverse reactions in the study group was lower (*P* < 0.05). The Hb levels, red blood cell counts, and HCT levels in the two groups were compared before and after blood transfusion. After blood transfusion, the Hb levels, red blood cell counts, and HCT levels of patients were all increased (*P* < 0.05). The levels of SPO2, Cr, and erythrocyte deformation index were compared before and after blood transfusion. Although the level of Cr decreased after blood transfusion, there exhibited no significant difference (*P* > 0.05). After blood transfusion, the SPO2 level and erythrocyte deformation index increased. Compared with the control group, the SPO2 level and erythrocyte deformation index in the study group were higher (*P* < 0.05). After blood transfusion, the levels of whole blood, red blood cells, and hemoglobin 2,3-DPG were all increased. The level of 2,3-DPG was higher compared to the control group (*P* < 0.05). The length of stay, hospital infection rate, and mortality after blood transfusion were compared. The average hospital stay was 18.36 ± 3.31 days in the study group and 32.87 ± 2.18 days in the control group; the length of stay in the study group was remarkably shorter (*P* < 0.05). Among them, 3 cases died in the study group, 1 case had nosocomial infection, 12 cases died in the control group, and 10 cases occurred nosocomial infection. The nosocomial infection rate and mortality in the study group were remarkably lower (*P* < 0.05). The above results show that the average hospitalization days of the study group are shorter, and the hospital infection rate and mortality are lower. The reason is that the study group improves the hypoxia state of patients' cells and tissues and then improves the therapeutic effect of patients.

Conclusively, with the extension of storage time, irreversible changes are taking place in red blood cells and their surrounding humoral environment, and these changes will have an important impact on the treatment process, outcome, and prognosis of patients with advanced malignant tumors. Compared with the risk of blood transfusion, the storage quality of red blood cells and the evaluation of curative effect after transfusion have been paid more and more attention. Effective blood transfusion is as important as safe transfusion. The purpose of this study is to provide some basis for clinical blood transfusion in the treatment of middle and advanced malignant tumor patients. It is suggested that personalized blood transfusion should be given to patients with advanced malignant tumor, and red blood cells with storage time ≤14 days should be infused as far as possible. This requires blood transfusion staff to further refine the management of blood storage, introducing a professional clinical blood transfusion management system, according to clinical diagnosis, disease characteristics, blood stock information, and diagnosis and treatment standards and guidelines.

## Figures and Tables

**Figure 1:** Overall survival curve of 120 patients with advanced cancer.

**Figure 2:** Comparison of total effective rate between the two groups.

**Figure 3:** Comparison of adverse reactions of blood transfusion between the two groups.

**Table 1:** General data of 120 dead patients.

Clinical parameter	Number of people	Constituent ratio (%)
Age (years)	63.15 ± 18.42	—
Gender		
Male	62	51.67
Female	58	48.33
Tumor type		
Lung cancer	21	17.50
Breast cancer	12	10.00
Digestive system tumor	52	43.33
Gynecological tumor	12	10.00
Urinary system tumor	8	6.67
Other tumors	15	12.50
Metastatic focus (unit)		
1 one	63	52.50
≥2 one	57	47.50
Transfer site		
Liver	45	37.50
Bone	44	36.67
Other	31	25.83
Surgical treatment		
Yes	64	53.33
No	56	46.67
Radiotherapy		
Yes	48	40.00
No	72	60.00
Chemotherapy		
Yes	71	59.17
No	49	40.83

**Table 2:** Univariate analysis of factors affecting survival of patients with advanced malignant tumor.

Factors	*N*	Percentage (%)	Average survival days	Median survival days	*P*
KPS					<0.05
<30	38	31.67	17 (13~21)	8 (6~10)	
≥30	82	68.33	29 (25~32)	20 (16~24)	
Dyspnea	0				<0.05
Yes	36	30.00	20 (14~25)	9 (7~11)	
No	84	70.00	27 (23~30)	19 (15~23)	
Delirium	0				<0.05
Yes	25	20.83	11 (7~15)	6 (4~8)	
No	111	92.50	28 (24~32)	21 (17~25)	
Red blood cell storage time (d)	0				<0.05
>14	51	42.50	20 (16~24)	18 (13~23)	
≤14	69	57.50	29 (24~33)	13 (7~19)	
Lym (%)	0				<0.05
≤12	78	65.00	22 (18~26)	13 (7~19)	
>12	42	35.00	30 (24~35)	25 (18~32)	
LDH (U/L)	0				<0.05
>500	50	41.67	17 (14~21)	9 (6~12)	
≤500	70	58.33	30 (25~34)	22 (17~27)	
ALB(g/L)	0				<0.05
<30	70	58.33	20 (16~24)	11 (7~15)	
≥30	50	41.67	31 (26~36)	26 (19~33)	

**Table 3:** Multivariate analysis of factors affecting survival of patients with advanced malignant tumor.

Variable	Univariate analysis (*P*)	Regression coefficient (*B*)	COXP	Relative risk exp (*β*)	95% confidence interval
KPS ≤ 20	<0.05	0.344	0.014	1.415	1.079~1.855
LDH > 500 U/L	<0.05	0.368	0.015	1.443	1.117~1.869
ALB < 30 g/L	<0.05	0.307	0.027	1.362	1.058~1.755
Delirium	<0.05	0.871	<0.001	2.388	1.684~3.387

**Table 4:** Comparison of DPG levels of whole blood, red blood cells, and hemoglobin in two groups before and after blood transfusion $\left[\bar{x}\pm s\right]$.

Hb (g/L)				Red blood cell count (×10^12^/L)		HCT (%)	

Group	*N*	Before blood transfusion	After blood transfusion	Before blood transfusion	After blood transfusion	Before blood transfusion	After blood transfusion
C group	36	61.18 ± 16.12	74.18 ± 15.32^a^	2.26 ± 0.64	3.86 ± 0.53^a^	17.24 ± 5.31	25.23 ± 5.51^a^
R group	36	62.38 ± 15.34	83.07 ± 17.37^b^	2.17 ± 0.69	5.01 ± 0.57^b^	17.07 ± 5.33	30.65 ± 5.76^b^
*t*		0.324	2.302	0.574	8.865	0.136	4.080
*P*		>0.05	<0.05	>0.05	<0.05	>0.05	<0.05

SPO_2_ (%)				Cr (*μ*mol/L)		Erythrocyte deformation index	

Group	*N*	Before blood transfusion	After blood transfusion	Before blood transfusion	After blood transfusion	Before blood transfusion	After blood transfusion
C group	36	82.53 ± 5.51	86.73 ± 4.81^a^	380.42 ± 292.25	330.93 ± 254.42^a^	0.75 ± 0.18	0.78 ± 0.14^a^
R group	36	81.97 ± 5.06	93.92 ± 4.41^b^	379.46 ± 291.55	328.15 ± 257.36^b^	0.74 ± 0.13	0.88 ± 0.11^b^
*t*		0.449	6.611	0.014	0.046	0.027	3.370
*P*		>0.05	<0.05	>0.05	>0.05	>0.05	<0.05

Whole blood (mmol/L)				Red blood cell (*μ*mol/ml)		Hemoglobin (*μ*mol/g)	

Group	*N*	Before blood transfusion	After blood transfusion	Before blood transfusion	After blood transfusion	Before blood transfusion	After blood transfusion
C group	36	2.11 ± 0.46	2.17 ± 0.24^a^	5.31 ± 0.92	6.03 ± 1.61^a^	16.17 ± 3.16	17.64 ± 5.18^a^
R group	36	2.13 ± 0.25	2.74 ± 0.45^b^	5.36 ± 1.04	7.68 ± 2.24^b^	16.82 ± 4.87	23.07 ± 5.63^b^
*t*		0.229	6.706	0.216	5.589	0.672	4.259
*P*		>0.05	<0.05	>0.05	<0.05	>0.05	<0.05

Note: comparison before and after blood transfusion in the control group, ^a^*P* < 0.05. Comparison of the study group before and after blood transfusion, ^b^*P* < 0.05.

## Data Availability

No data were used to support this study.
